# Relationship between the Quantitative Indicators of Cranial MRI and the Early Neurodevelopment of Preterm Infants

**DOI:** 10.1155/2021/6486452

**Published:** 2021-11-19

**Authors:** Jing Yin, Yanhui Wu, Yuxuan Shi, Lu Shen, Qigai Yin

**Affiliations:** ^1^Department of Pediatrics, Xuzhou Medical University Affiliated Hospital of Lianyungang, Lianyungang 222000, China; ^2^Department of Pediatrics, Lianyungang Clinical Medical College of Nanjing Medical University, Lianyungang 222042, China

## Abstract

**Aim:**

To explore the relationship between the quantitative indicators (biparietal width, interhemispheric distance) of the cranial MRI for preterm infants at 37 weeks of postmenstrual age (PMA) and neurodevelopment at 6 months of corrected age.

**Methods:**

A total of 113 preterm infants (gestational age < 37 weeks) delivered in the Obstetrics Department of the First People's Hospital of Lianyungang from September 2018 to February 2020 and directly transferred to the Neonatology Department for treatment were enrolled in this study. Based on their development quotient (DQ), the patients were divided into the normal (DQ ≥ 85, *n* = 76) group and the abnormal (DQ < 85, *n* = 37) group. Routine cranial MRI (cMRI) was performed at 37 weeks of PMA to measure the biparietal width (BPW) and interhemispheric distance (IHD). At the corrected age of 6 months, Development Screening Test (for children under six) was used to assess the participants' neurodevelopment.

**Results:**

Univariate analysis showed statistically significant differences in BPW, IHD, and the incidence of bronchopulmonary dysplasia between the normal and the abnormal groups (*P* < 0.05), while no statistically significant differences were found in maternal complications and other clinical conditions between the two groups (*P* > 0.05). Binary logistic regression analysis demonstrated statistically significant differences in IHD and BPW between the normal and the abnormal groups (*95% CI*: 1.629-12.651 and 0.570-0.805, respectively; *P* = 0.004 and *P* < 0.001, respectively), while no significant differences were found in the incidence of bronchopulmonary dysplasia between the two groups (*95% CI:* 0.669-77.227, *P* = 0.104). Receiver operating characteristic curve revealed that the area under the curve of BPW, IHD, and the joint predictor (BPW + IHD) were 0.867, 0.805, and 0.881, respectively (*95% CI*: 0.800-0.933, 0.710-0.900, and 0.819-0.943, respectively; all *P* values < 0.001).

**Conclusion:**

BPW and IHD, the two quantitative indicators acquired by cMRI, could predict the neurodevelopmental outcome of preterm infants at the corrected age of 6 months. The combination of the two indicators showed an even higher predictive value.

## 1. Introduction

Postpartum depression (PPD) affects approximately 10–15% of women and is one of the most common complications of child-bearing [1]. The consequences of PPD for both mother and infant are well established: women who suffer from PPD are twice as likely to experience future episodes of depression over a 5-year period. PPD can also impair maternal–infant interactions, leading to attachment insecurity, developmental delay, and social interaction difficulties in affected children. Late (34-36 weeks' gestational age) and moderate (32-33 (6/7) weeks' gestational age) preterm infants constitute approximately 84% of all preterm infants. Over the past few decades, there is increasing recognition that this population is at risk for short- and long-term morbidities and adverse outcomes [1, 2]. The survival rate of preterm infants has been significantly increased with the advancement of medical technologies. Recent data from several sources indicate improvements in survival for extremely preterm (EPT) infants in the US and other international developed nations. Based on estimates from the Neonatal Research Network (NRN), 74% of EPT infants survive the initial birth hospitalization, although each decreasing gestational age (GA) week has substantial effects on mortality, particularly for infants born at 22-25 weeks GA [2]. But due to the immature structural development, the preterm infants face various challenges and risks after birth, among which the neurodevelopmental dysplasia caused by brain injury has always been the focus of people's attention. Imaging technology has confirmed that the poor neurodevelopmental outcome of preterm infants can be attributed to intracranial hemorrhage [1, 2], periventricular-intraventricular hemorrhage with ventricular enlargement [3], abnormal white matter [4–7], etc. However, macroscopic brain damage shown on cranial magnetic resonance imaging (cMRI) cannot fully demonstrate the neurodevelopmental outcome. Therefore, to comprehensively predict the neurodevelopmental outcome, Kidokoro et al. [8] proposed a new scoring method for cMRI, which could not only qualitatively assess brain injury but also quantitatively analyze the maturity of brain development using indicators like the interhemispheric distance (IHD) and biparietal width (BPW) [9]. To the best of our knowledge, few studies have focused on the relationship between the quantitative assessment of premature infants' brain development and neurodevelopmental outcome. By exploring the relationship between IHD, BPW, and the neurodevelopmental prognosis of preterm infants at a corrected age of 6 months, this study is aimed at finding quantitative indicators of cMRI that could predict the prognosis of early neurodevelopment for early identification and intervention of adverse neurodevelopmental outcome in high-risk infants.

## 2. Methods

### 2.1. Participants

A total of 496 preterm infants (gestational age < 37 weeks) delivered in the Obstetrics Department of the First People's Hospital of Lianyungang from September 2018 to February 2020 were initially enrolled. Among them, 324 completed cMRI at 37 weeks of postmenstrual age (PMA), and 156 cases completed the Developmental Screening Test (DST) for children under six at 6 months of corrected age. Finally, the clinical data of 113 preterm infants were analyzed and researched. Informed consents were obtained from the infants' parents, and the ethics committee of The First People's Hospital of Lianyungang approved this study (ethics review number: KY20181102001). The inclusion criteria were as follows: gestational age (GA) < 37 weeks, regular obstetric check-ups in the Obstetrics Department of our hospital during pregnancy, and complete clinical data of pregnant mothers and preterm infants. The exclusion criteria were as follows: congenital malformations; genetic metabolic diseases; asphyxia, convulsions, hypoxic-ischemic encephalopathy (HIE), high bilirubin encephalopathy, and other high-risk factors that cause abnormal brain function; brain injury such as intracranial hemorrhage and abnormal white matter found by cranial ultrasound or cMRI examination; and death or failure to meet clinical discharge standards and treatment abandonment by parents.

### 2.2. Clinical Data

The clinical data of 113 premature infants and their mothers were collected, including gender, number of fetuses, delivery method, pregnancy method, hospitalization time, GA, birth weight (BW), head circumference, height, oxygen inhalation time, antenatal corticosteroids (ACS), wet lung, respiratory distress syndrome (RDS), bronchopulmonary dysplasia (BPD), pneumonia, jaundice, retinopathy of prematurity (ROP), necrotizing enterocolitis (NEC), gestational diabetes mellitus (GDM), gestational hypertension (GH), anemia during pregnancy, premature rupture of fetal membranes, placental abruption, and placenta previa.

### 2.3. Developmental Outcome

The neurodevelopment of the preterm infants at 6 months of corrected age was assessed using DST in the Child Care Outpatient Department of our hospital. DST, revised based on Denver Mental Development Screening Method and compiled by The Pediatric Hospital Affiliated to Fudan University, included 120 items on mental and motor abilities and social adjustment abilities targeting children aged 0-6 years. Being efficient and easy to operate, DST showed good reliability and validity. The test results of DST were presented as a development quotient (DQ) and mental index. Based on DQ, children under 3 years old were classified into three grades: abnormal (DQ < 70), suspicious (DQ between 70 and 84), and normal (DQ ≥ 85). In this study, suspicious and abnormal children fell into the group of abnormal neurodevelopment and those with DQ ≥ 85 into the group of normal neurodevelopment.

### 2.4. cMRI

cMRI was performed using American GE (Signa HDxt) 1.5T instrument at 37 weeks of PMA. The parameters of cMRI scan were as follows: T2 fast spin echo (FSE) sequence, radio frequency pulse repetition time (TR) = 3000 ms, and echo time (TE) = 85 ms. The T1WI parameters were as follows: TR 1750 ms, TE = 24 ms, field of view (FOV) 24 cm, layer thickness 5 mm, and no spacing. The T2WI sequence parameters were as follows: TR = 8500 ms, TE = 155 ms, FOV = 24 cm, layer thickness 5 mm, and no spacing. The T2 coronal position was selected to measure the BPW and IHD with bilateral cochlea and base as the standard. BPW was defined as the maximum horizontal width of the frontal lobe; IHD was defined as the horizontal distance between the top of the frontal gyri of the two cerebral hemispheres (Figure 1). All preterm infants were given intravenous injection of phenobarbital sodium (5 mg/kg) 30 minutes before the cMRI examination and wrapped with a cotton quilt. The examination was performed when the infants were asleep. All cMRI data were acquired and recorded by two radiologists without knowledge of the clinical situation.

### 2.5. Statistical Analysis

The SPSS 25 software was used for statistical analysis. For univariate analysis, nonnormally distributed continuous variables were presented as M (Q1-Q3). Mann–Whitney *U* test was used for between-group comparison. Normally distributed continuous variables were presented as mean ± standard deviation. Two independent sample *t*-test was used for comparison between groups. Enumeration data were expressed as examples. The Chi-square test, *t*-test, and *Mann–WhitneyU* test were used to perform univariate analysis on the clinical data of the participants. Binary logistic regression was selected for multivariate analysis, and receiver operating characteristic curve was used to evaluate the value of BPW and IHD in predicting the early neurodevelopmental outcome of preterm infants. The receiver operating characteristic curve (ROC) was used to analyze the variables with *P* < 0.05 in multivariate analysis. A *P* value < 0.05 was considered significant.

## 3. Results

A total of 113 preterm infants were enrolled, including 76 in the normal group and 37 in the abnormal group. As shown in Table 1, the IHD of the normal group was smaller than that of the abnormal group (3.0 mm vs. 3.8 mm), and the BPW of the normal group was larger than that of the abnormal group (72.8 mm vs. 66.6 mm). The differences were statistically significant (*P* < 0.05). There was no significant difference in the other general conditions between the two groups (*P* > 0.05) (Table 1).

### 3.1. Comparison of Complications

As shown in Table 2, the incidence of BPD was lower in the normal group than the abnormal group (1.3% vs. 13.5%), and the difference was statistically significant (*P* < 0.05). There was no statistically significant difference in maternal and other complications of preterm infants between the two groups (*P* > 0.05) (Table 2).

### 3.2. Multiple-Factor Analysis

Binary logistic regression model was used to further analyze the variables with single factor *P* < 0.05. The results showed that BPD was not an independent risk factor for DST abnormality (*OR*: 7.186, *95% CI*: 0.669-77.227, *P* = 0.104). Both IHD and BPW were independent predictors of DST abnormality (*OR* values: 4.540, 0.677; *95% CI*: 1.629-12.651, 0.570-0.805; *P* values: both < 0.05). The details are shown in Table 3.

### 3.3. Predictive Value of Different Variables on Neurodevelopmental Outcome

ROC curve results showed that the area under the curve (AUC) of the combined predictor (IHD + BPD), BPW, and IHD were 0.881 (*95% CI*: 0.819-0.943, *P* < 0.001), 0.867 (*95% CI*: 0.800-0.933, *P* < 0.001), and 0.805 (*95% CI*: 0.710-0.900, *P* < 0.001), respectively. The value of the combined predictor (IHD + BPW) in predicting neurodevelopmental abnormalities was higher than that of BPW or IHD alone. The maximum Youden index of the combined predictor (IHD + BPW) was 0.668, the sensitivity was 0.892, and the specificity was 0.776. The details are shown in Figure 2.

## 4. Discussion

The third trimester of pregnancy is essential for the development of the fetal brain. However, due to early separation from the protective environment in utero and early exposure to the outside world, premature infants are prone to brain damage and neurodevelopmental diseases after birth, such as cerebral palsy, intellectual impairment, cognitive deficiency, and developmental delay [10]. The cMRI results have shown that 50% to 80% of very preterm infants have diffuse white matter abnormalities [11]. Preterm infants with obvious abnormal cMRI results can be monitored closely for neurodevelopmental abnormalities and receive prompt intervention. However, in clinical practice, the neurodevelopmental abnormalities in premature infants with atypical brain injury symptoms and no abnormal cMRI results are often ignored. Thus, the lagged manifestations of nervous system injury may delay treatment and impair their health. In a study on preterm infants with a GA of 24-32 weeks, Chau et al. [12] found that even if no abnormal changes (such as cerebral hemorrhage and white matter abnormality) were observed in cMRI, motor development retardation could appear at 18 months after birth. Therefore, early identification and intervention of preterm infants at risk of neurodevelopmental abnormalities are essential for their quality of life. So far, few studies have combined quantitative cMRI indicators with neurodevelopmental tests to evaluate the brain development of preterm infants. The present study is aimed at finding an objective quantitative cMRI indicator to detect the abnormal brain development of preterm infants at an early stage. In this study, two quantitative indicators of cMRI, BPW and IHD, were selected to evaluate brain development, and the association of these two indicators with early neurodevelopmental outcome of premature infants was studied. BPW can indicate the volume of brain white matter and the absolute size of the brain, while IHD demonstrates the development of brain gray matter and the brain growth restriction relative to the head circumference. Using these two quantitative indicators to evaluate brain growth and development can further clarify the influence of brain structure on brain function.

The results of this study showed smaller IHD and larger BPW in the normal group than the abnormal group, and the differences were statistically significant (*P* < 0.05). Binary logistic regression analysis revealed that larger IHD was an independent risk factor for neurodevelopmental abnormalities (*OR* 4.540, *95% CI* 1.629-12.651, *P* = 0.004), while larger BPW was an independent protective factor for neurodevelopmental abnormalities (*OR* 0.677, *95% CI* 0.570-0.805, *P* < 0.001). The ROC curve suggested that the combination of IHD and BPW had a higher value in predicting neurodevelopmental abnormality. The AUC of the combined predictor (IHD + BPW), BPW, and IHD was 0.881, 0.867, and 0.805, respectively. The follow-up study on the relationship between BPW, IHD, and the neurodevelopmental outcome in preterm infants by Kidokoro et al. [13] demonstrated that a smaller BPW was associated with cognitive developmental delay at 2 years of age as assessed by the Bayley scale. Hüning et al. [14] studied preterm infants with GA < 32 weeks and found that IHD could predict the neurodevelopmental outcome of preterm infants at 2 years of age. The studies by Tich et al. [15] and Dewan et al. [16] showed that BPW was related to the neurodevelopmental prognosis of preterm infants at 24 months of corrected age. The results of our study were consistent with the abovementioned studies. Our results also revealed that the IHD ((3.0 or 3.8) mm) of premature infants at 37 weeks of gestational age was relatively larger, and the BPW ((72.8 or 66.6) mm) was relatively smaller. Yet, in the study by Walsh et al. [17], BPW was larger (83.6 ± 4.4 mm), and IHD was smaller (2.5 ± 1.2 mm) in preterm infants at 41.5 ± 1.2 weeks of PMA with an average GA of 34.4 ± 1.2 weeks, compared with the results of our study. This difference might be caused by the difference in time when cMRI was performed. In our study, the cMRI scan was conducted at 37 weeks of PMA. Based on cMRI scan results, Kidokoro et al. [8] found that compared with term infants, the overall brain measurements of premature infants were smaller, and there was a linear relationship between BPW, IHD, and the corrected GA. In this study, the cMRI scans of preterm infants at 36-42 weeks of PMA showed that the average values of BPW and IHD in preterm infants and term infants were 72.4 mm vs. 81.7 mm and 3.6 mm vs. 2.6 mm, respectively. This difference further reveals the constantly changing brain volume of premature infants: BPW gradually increases, and IHD gradually decreases as GA increases.

Since this study only involved the cMRI data of preterm infants, the IHD and BPW data of preterm and term infants were not compared. Therefore, the IHD and BPW data of preterm infants and term infants were not further compared. The study by Walsh et al. [17] showed compared with preterm infants, BPW of term infants was larger, and IHD was smaller than those of Brumbaugh et al. [18] reported that the overall brain volume of premature infants was smaller than that of term infants, and this structure could impact cognition, memory, and processing speed of premature infants at the age of 6-13 years. At the same time, another shortcoming of this study was that cMRI scans were not performed in the preterm infants immediately after birth, so a longitudinal comparison of IHD and BPW could not be completed. George et al. [19] found a higher association of MRI results at premature infant period with the cognitive function of preterm infants at 12 months of correction compared with motor function. Gui et al. [20] showed that the qualitative MRI measurement values at birth and at term of corrected gestational age were correlated with the motor outcome at corrected gestational age of 18-24 months, and the brain tissue volume at term was correlated with the cognitive outcome at 5 years of age.

Due to the immature development, the premature infants were prone to brain damage after birth. Despite normal brain development as revealed by head ultrasound and cMRI, these infants may still suffer neurodevelopmental disorders in the later stage of life [21], which is probably related to the subtle differences in brain structure [22]. At present, though diffusion-tensor imaging (DTI) and magnetic resonance spectroscopy (MRS) can be used to perform subtle evaluation of brain microstructure [12, 23–25], the high requirements of DTI and MRS preclude their wide implementation in primary hospitals. In our study, the measurement of IHD and BPW was performed using cMRI, which is more operatable and accessible for most clinicians. Our results showed that IHD and BPW could be used as early predictors of neurodevelopmental prognosis, and the combined predictor (IHD + BPW) showed an even greater value in predicting DST abnormalities. However, this study is not polycentric. Therefore, multicenter studies with large sample sizes are needed to determine the relationship between the predictors and neurodevelopmental abnormality in order to maximize their predictive potentials and improve the prognosis of preterm infants.

## Figures and Tables

**Figure 1:** cMRI. Routine cranial MRI (cMRI) was performed at 37 weeks of PMA to measure the BPW and IHD. All preterm infants were given intravenous injection of phenobarbital sodium (5 mg/kg) 30 minutes before the cMRI examination and wrapped with a cotton quilt. The examination was performed when the infants were asleep. All cMRI data were acquired and recorded by two radiologists without knowledge of the clinical situation. IHD: interhemispheric distance; BPW: biparietal width.

**Figure 2:** The ROC curve of the combined predictor (BPW + IHD), IHD, and BPW in predicting abnormal neurodevelopment. ROC: receiver operating characteristic curve. The maximum Youden index of the combined predictor (IHD + BPW) was 0.668, the sensitivity was 0.892, and the specificity was 0.776.

**Table 1:** Comparison of general data of preterm infants.

	Normal (76)	Abnormal (37)	*χ* ^2^/*z*/*t*	*P*
Male	46 (60.5)	19 (51.4)	0.857	0.354
Singleton pregnancy	58 (76.3)	30 (81.1)	0.328	0.567
Vaginal delivery	18 (23.7)	7 (18.9)	0.328	0.567
Natural pregnancy	68 (89.5)	33 (89.2)	0.002	0.963^∗^
ACS	49 (64.5)	22 (59.5)	0.268	0.605
Hospitalization time (d)	13 (10-19.5)	14 (11.5-22.0)	-0.589	0.556
GA (w)	34.9 (33.7 ± 36.1)	35.1 (33.7 ± 35.8)	-0.150	0.881
BW (g)	2375.0 (1985.0-2637.5)	2390.0 (1865.0-2730.0)	-0.089	0.929
Height (cm)	47.0 (45.0-48.0)	46.5 (44.0-48.5)	-0.600	0.570
Head circumference (cm)	32.0 (30.0-33.0)	32.5 (31.0-33.3)	-0.559	0.576
Oxygen inhalation time (d)	1.0 (0.0-4.0)	2.0 (1.0-3.5)	-0.789	0.425
IHD (mm)	3.0 (2.6-3.5)	3.8 (3.5-4.2)	-5.254	<0.001
BPW (mm)	72.8 ± 4.2	66.6 ± 3.8	7.689	<0.001

^∗^Continuity correction. ACS: antenatal corticosteroids; GA: gestational age; BW: birth weight; IHD: interhemispheric distance; BPW: biparietal width.

**Table 2:** Comparison of complications between normal and abnormal groups.

	Normal (76)	Abnormal (37)	*χ* ^2^	*P*
Wet lung	4 (5.3)	6 (16.2)	2.468	0.116^①^
RDS	13 (17.1)	5 (13.5)	0.240	0.624
BPD	1 (1.3)	5 (13.5)	5.138	0.023^①^
Pneumonia	25 (32.9)	12 (32.4)	0.002	0.961
Jaundice	56 (73.7)	24 (64.9)	0.936	0.333
ROP	1 (1.3)	3 (8.1)	1.667	0.197
NEC	2 (2.6)	0 (0.0)	—	1.000^②^
GDM	14 (18.4)	4 (10.8)	1.076	0.300
GH	21 (27.6)	13 (35.1)	0.666	0.414
Anemia during pregnancy	8 (10.5)	3 (8.1)	0.005	0.945
Premature rupture of fetal membranes	24 (31.6)	11 (29.7)	0.400	0.842
Placental abruption	2 (2.6)	1 (2.7)	<0.001	1.000^①^
Placenta previa	7 (9.2)	4 (10.8)	<0.001	1.000^①^

① Continuity correction; ② Fisher's exact test. RDS: respiratory distress syndrome; BPD: bronchopulmonary dysplasia; ROP: retinopathy of prematurity; NEC: necrotizing enterocolitis; GDM: gestational diabetes mellitus; GH: gestational hypertension.

**Table 3:** Results of logistic regression analysis.

Factors	*B*	S.E.	Wald	Exp	95% CI	*P*
IHD (mm)	1.513	0.523	8.370	4.540	1.629-12.651	0.004
BPW (mm)	-0.390	0.088	19.513	0.677	0.570-0.805	<0.001
BPD	1.972	1.212	2.649	7.186	0.669-77.227	0.104

IHD: interhemispheric distance; BPW: biparietal width; BPD: bronchopulmonary dysplasia.

## Data Availability

The authors confirm that the data supporting the findings of this study are available within the article.
